The article "The Effects of Chinese Herbal Decoction Combined with Recombinant Human Interferon α2b on MRI Imaging, Tumor Markers, and Immune Function in Patients with Renal Cell Carcinoma" was published in 2021. Journal: Evid Based Complement Alternat Med.

# The Effects of Chinese Herbal Decoction Combined with Recombinant Human Interferon *α*2b on MRI Imaging, Tumor Markers, and Immune Function in Patients with Renal Cell Carcinoma

**DOI:** 10.1155/2021/8106974

**Published:** 2021-10-25

**Authors:** Siliang Song, Wen Li, Wenjuan Liang, Xiu Tian

**Affiliations:** ^1^Department of Imaging, Qingdao Hospital of Traditional Chinese Medicine, Qingdao Hiser Hospital, Qingdao 266033, Shandong, China; ^2^Department of Radiotherapy, Qingdao Hospital of Traditional Chinese Medicine, Qingdao Hiser Hospital, Qingdao 266033, Shandong, China

## Abstract

**Background:**

To explore the clinical efficacy of traditional Chinese medicine decoction combined with recombinant human interferon *α*2b in the treatment of renal cell carcinoma (RCC).

**Methods:**

68 RCC patients were divided into the control group and treatment group (*n* = 34). The control group was treated with recombinant human interferon *α*2b, and the treatment group was treated with traditional Chinese medicine decoction on the basis of the control group. The clinical efficacy and life quality were observed. At the same time, the changes of immune function before and after treatment were compared.

**Results:**

After one course of treatment, the effective rate and clinical benefit rate of the treatment group were higher than those of the control group. The Karnofsky score in the treatment group was better than that in the control group. In improving the immune function, the treatment group was better than the control group in increasing CD3+ and CD4+ and reducing CD8+.

**Conclusion:**

Traditional Chinese medicine decoction combined with recombinant human interferon *α*2b has a good effect on the treatment of RCC. It can not only improve the common clinical symptoms of patients but also improve the quality of life and cellular immune function of patients.

## 1. Introduction

Renal cell carcinoma (RCC) is one of the common malignant tumors in the urinary system. Its incidence accounts for about 3% of clinical cancer patients [1–3], and it is increasing year by year. The etiology of RCC is not clear and may be related to smoking, obesity, and hypertension [4]. Clinically, patients with low back pain, hematuria, and abdominal masses are typical symptoms, which may be accompanied by hypertension, fever, anemia, and abnormal coagulation function [5, 6]. There are no obvious symptoms in the early stage of RCC. When there are obvious symptoms, a small number of patients have lesions confined to the kidneys. Most patients have unpredictable metastases. Metastatic RCC seriously affects the life quality of patients, and its therapeutic effect and prognosis are not ideal. Moreover, RCC is not sensitive to radiotherapy and chemotherapy but is more sensitive to immunotherapy and targeted therapy [7].

The article "The Effects of Chinese Herbal Decoction Combined with Recombinant Human Interferon α2b on MRI Imaging, Tumor Markers, and Immune Function in Patients with Renal Cell Carcinoma" was published in 2021. Journal: Evid Based Complement Alternat Med.

At present, the modern medical treatment of RCC is mainly based on radical nephrectomy [8–12], postoperative adjuvant targeted therapy, and immunotherapy. However, targeted therapy and immunotherapy are expensive and have large side effects, which cannot effectively delay disease progression [13]. The long-term effect is not good. In the past 20 years, the 5-year survival rate of patients with advanced RCC has been very low. The main reason is the lack of effective treatments. Clinically, most advanced RCC have metastasized far away and cannot be treated with surgery. Although immunotherapy and targeted therapy have certain short-term effects, they have serious side effects and poor long-term effects [14]. The clinical effect of the combination of Chinese and Western medicine in the treatment of RCC is better. The multifaceted and multilayered mechanism reflects the unique advantages of Chinese medicine. Previous studies have shown that [15–18] TCM adjuvant therapy emphasizes syndrome differentiation and has multilevel, multitarget, and multidirectional effects. Adjuvant treatment of Chinese medicine has a positive effect on improving clinical symptoms, improving immunity, reducing toxicity, improving life quality, preventing recurrence and metastasis, and prolonging survival time.

Surgery is currently the most effective way to treat RCC. At the same time, interferon adjuvant therapy should be given to patients with RCC [19]. Interferon *α*2b has obvious antitumor effects, which can inhibit cell proliferation and improve the immune function [16]. After interferon *α*2b binds to the cell surface receptors, it can significantly improve the immune function and enhance the phagocytosis of macrophages. It can also accelerate the apoptosis of cancer cells and exert a powerful inhibitory effect. However, patients often have symptoms, such as fever, chills, body aches, cytopenias, nausea, and indigestion after the application of interferon [20]. This will lead to interferon reduction or even discontinuation, thereby affecting the standard treatment of RCC patients.

In view of this, patients were given the adjuvant therapy of recombinant human interferon *α*2b combined with Chinese medicine decoction. This study aimed to explore the effects of recombinant human interferon *α*2b combined with Chinese medicine decoction on MRI imaging manifestations, tumor markers and immune function in patients with RCC.

## 2. Materials and Methods

### 2.1. Clinical Data

This study is a retrospective study. The cases were all RCC patients who were admitted to Qingdao Hospital of Traditional Chinese Medicine, Qingdao Hiser Hospital from January 2019 to December 2020. 71 RCC patients who met the criteria were selected and all met the relevant diagnostic criteria for renal cancer in the “practical oncology.” Renal surgery specimens were confirmed by cytopathology or histopathology. Examinations, such as abdominal MRI, CT, or PET-CT, showed the existence of space-occupying lesions. Patients has typical clinical manifestations, such as hematuria, abdominal masses, and waist and abdomen pain. The age of the patients was 18 to 75 years old. Physical status Karnofsky (KPS) score was ≥60 points. Patients did not receive other antibell tumor treatment one month before the experiment. All patients voluntarily signed informed consent forms. This study was approved by the Institutional Ethics Committee of Qingdao Hospital of Traditional Chinese Medicine, Qingdao Hiser Hospital. Patients with metastatic RCC, severe liver, cardiovascular and hematopoietic system, and other primary diseases, patients receiving other treatments, psychiatric patients, patients with obvious bleeding tendency and severe electrolyte disorders, patients with immunotherapy contraindications, patients with allergic physique, and pregnant or lactating women were excluded from this study.

The article "The Effects of Chinese Herbal Decoction Combined with Recombinant Human Interferon α2b on MRI Imaging, Tumor Markers, and Immune Function in Patients with Renal Cell Carcinoma" was published in 2021. Journal: Evid Based Complement Alternat Med.

Case rejection and dropout were as follows. After inclusion, those cases that did not meet the inclusion criteria or did not use the drugs according to the experimental protocol should be eliminated. The included cases that have serious adverse events or complications and are not suitable for continuing to accept the experimenter, withdrawing by themselves, or failing to complete the entire treatment process shall be regarded as dropped cases. Those that fail to check in accordance with regulations or whose main indicators are missing shall be eliminated.

According to the case rejection and dropout criteria, 68 cases finally completed the entire treatment process. There was no significant difference in staging between the two groups. According to the treatment method, the patients were divided into a control group and a treatment group, with 34 cases in each group. General data balance test is shown in Table 1.

As shown in Table 1, gender, age, Karnofsky score, tumor location, Robson tumor stage, and case classification were all *P* > 0.05 between the two groups. It indicates that there is no significant difference between the two groups of data, and the data are well balanced and comparable.

### 2.2. Treatment Methods

Patients in the control group were injected subcutaneously with recombinant human interferon *α*2b. The dosage is 3 million IU/day × 2 weeks (1–2 weeks), 6 million IU/day × 2 weeks (3–4 weeks), and 9 million IU/day × 2 weeks (5–6 weeks). Six weeks is a course of treatment, and all patients are treated for 1 course.

The article "The Effects of Chinese Herbal Decoction Combined with Recombinant Human Interferon α2b on MRI Imaging, Tumor Markers, and Immune Function in Patients with Renal Cell Carcinoma" was published in 2021. Journal: Evid Based Complement Alternat Med.

The treatment group was treated with Lishen Huazhuo Decoction on the basis of the control group. Lishen Huazhuo Decoction contains 30 g of Salvia miltiorrhiza, 30 g of Chinese yam, 20 g of cattail yellow, 15 g of malt, 15 g of Taizi ginseng, 15 g of *Pteris vulgaris*, 10 g of *Ulmus pumila*, 10 g of *Imperata* root, 10 g of licorice, and 3 g of rhubarb. Lishen Huazhuo Decoction was prepared according to the above ratio (1 dose/d). During the medication period, the diet should be strictly in accordance with the doctor's advice, fasting spicy, and irritating food.

### 2.3. MR Inspection Method

Patients fasted for 4 h before the MR examination. Before the patient enters the scanning room, all metal materials outside the body should be removed. It should be confirmed that there are no contraindications to MR examination. All patients took the supine position and received end-inspiratory breath-holding and breathing amplitude consistency training.

Siemens SKYRS 3.0T MR scanner is used for MR inspection. The patient is in the supine position, and an end-inspiratory breath-hold scan is performed to keep the baseline level of each sequence the same. The scan range includes all kidneys. After the regular scan is completed, a dynamic enhanced scan is performed. The conventional scanning sequence includes axial T2WI, axial T2WI fat suppression sequence, coronal T2WI, and axial T1WI (positive phase, reverse phase). The layer thickness of the axial T12WI, T2WI, and T2WI fat suppression sequence is 5.0 mm, and the layer spacing is 1.1 mm. The layer thickness of coronal T2WI is 6.0 mm, and the layer spacing is 1.0 mm. Multiphase dynamic enhancement scanning adopts three-dimensional volume interpolation fast spoiling VIBE (GRE T1WI) technology. Scans of early medullary cortex, late cortex medulla, renal parenchymal phase, and excretory phase were performed at 20–30 s, 45–70 s, 100–260 s, and 200–360 s after the injection of the contrast agent. The contrast agent Gd-DTPA injection should be injected through the cubital vein with a high-pressure syringe at a speed of 2.5 ml/s, with a dose of 0.1 mmol/kg. After the contrast agent is injected, 20 ml of normal saline was added.

### 2.4. MR Image Analysis and Data Processing

The images are observed and analyzed by two experienced MR diagnostic physicians. When there is a disagreement on the analysis results, two MR diagnostic physicians negotiate and reach a consensus. The main analysis included the following: (1) the location of the lesion, (2) signal characteristics, which compared with normal renal parenchyma, is divided into low signal, low signal-based mixed signal, high-level low-mix signal, and high signal-based mixed signal and high signal, (3) edge condition, which should confirm whether there is a thin ring high (low) signal or whether there is a nodular or irregular shape abnormal signal, and (4) the characteristics of dynamic strengthening, which are divided into no strengthening, ring-shaped strengthening, irregular edge shape, and nodular strengthening. Compared with the renal cortex, the degree of enhancement is divided into obvious enhancement, moderate enhancement, and mild enhancement.

The article "The Effects of Chinese Herbal Decoction Combined with Recombinant Human Interferon α2b on MRI Imaging, Tumor Markers, and Immune Function in Patients with Renal Cell Carcinoma" was published in 2021. Journal: Evid Based Complement Alternat Med.

### 2.5. Observation of Curative Effect

#### 2.5.1. Short-Term Objective Curative Effect (Solid Tumor Size)

According to the latest evaluation standards for the efficacy of solid tumors, the short-term efficacy evaluation of renal cancer is divided into complete remission (CR), partial remission (PR), stable (SD), and progress (PD). The short-term curative effect CR + PR is defined as effective. The percentage of all cases that can be evaluated is effective rate. The solid tumor of kidney cancer was selected as the measurement lesion, and the lymph node, bone, liver, or lung metastasis lesions were not used as the measurement lesion. ① Complete remission is as follows: it can be seen that the tumor lesions disappeared completely and remained for more than 4 weeks. ② Partial remission is as follows: the maximum diameter of the tumor lesion has been reduced by ≥50%. No new lesions appeared, which maintained for more than 4 weeks. ③ Stable cases are as follows: the maximum diameter of the tumor lesion is reduced by less than 25% or increased by no more than 50%. No new lesions appeared, which maintained for more than 4 weeks. ④ Progress is as follows: the maximum diameter of tumor lesions increased by ≥20% or new lesions appeared.

#### 2.5.2. Improvement of Common Clinical Symptoms

The clinical effect of patients is divided into three categories: improvement, stability, and ineffectiveness. According to the standards of “Guiding Principles for Clinical Research of New Chinese Medicines (Practice),” the efficacy of patients is identified. Among them, there are five standard test indicators, such as fatigue, dry mouth and throat, lumbar muscle soreness, five upset and hot, and abnormal stool. Each indicator includes 0 to 3 points. Improvement means that the score after treatment is 0–30% of that before treatment. Stable means that the score after treatment is 30% to 70% of that before treatment. Invalid means that the score after treatment is 70% to 100% of the score before treatment. The total effective rate is the ratio of (improvement + stability) to the total effective rate.

The article "The Effects of Chinese Herbal Decoction Combined with Recombinant Human Interferon α2b on MRI Imaging, Tumor Markers, and Immune Function in Patients with Renal Cell Carcinoma" was published in 2021. Journal: Evid Based Complement Alternat Med.

#### 2.5.3. Quality of Life

Quality of life is evaluated once before and after treatment. The KPS physical status scoring standard is used to evaluate and record the quality of life (QOL). ① Improvement means that the KPS value increased by >10 points. ② Stability means that the fluctuation range of KPS value <10 points. ③ Decrease means that the KPS value decreased by >10 points:

(1) $$\begin{array}{c} \text{improvement rate}=\frac{\left(\text{improvement}+\text{stability}\right)}{\text{total number of cases}}. \end{array}$$

### 2.6. Index Measurement

#### 2.6.1. Changes in Cellular Immune Function (CD3+, CD4+, CD8+, and CD4+/CD8+) before and after Treatment (Flow Cytometry)

Before and after treatment, 5 mL of fasting venous blood was drawn from the patient and centrifuged in an automatic blood centrifuge. The centrifuge speed was adjusted to 3000 r/min and centrifuged for 10 min. The supernatant was taken and placed in a refrigerator at −20°C for inspection. Flow cytometry was used to detect the relevant indicators of T lymphocyte subsets in serum. CD3+, CD4+, CD8+, and other T lymphocyte subsets were detected by Beckman Coulter EpicsXL flow cytometer.

#### 2.6.2. Detection of Tumor Markers (Electrochemiluminescence Immunoassay)

Enzyme-linked immunoassay was used to determine the levels of neuron-specific enolase (NSE), carcinoembryonic antigen (CEA), human *β*2 microglobulin (*β*2-MG), and ferritin (FERR) tumor markers before and after treatment.

### 2.7. Observation Time

1. Symptoms and signs are recorded once a week
2. Imaging tumor examination (MRI) was performed before treatment and once after the end of the first course of treatment

### 2.8. Statistical Analysis

SPSS 22.0 statistical analysis software was used to process and analyze the data. The measurement data is described by the mean ± standard deviation, and the independent sample *t*-test is selected for comparison. The count data is expressed as a ratio or percentage (%), and the comparative analysis was performed by chi-square test. The difference was statistically significant at *P* < 0.05.

## 3. Results

### 3.1. MRI Features before and after Treatment

Among the 34 cases in the control group, MRI judged 10 cases of septal thickening (cancer wall thickness, 2.89 ± 0.70 mm), 16 cases of calcification, and 8 cases of solid component. MRI T1WI examination showed that 27 cases had clear boundary and 7 cases had blurred boundary. T2WI showed 26 cases of high signal, 5 cases of slightly high signal, and 3 cases of equal signal. Among the 34 patients in the treatment group, MRI judged 11 cases of septal thickening (cancer wall thickness, 2.86 ± 0.56 mm), 17 cases of calcification, and 6 cases of solid component. MRI T1WI examination showed that 28 cases had clear borders and 6 cases had blurred borders. T2WI showed 25 cases of high signal, 6 cases of slightly high signal, and 3 cases of equal signal.

The article "The Effects of Chinese Herbal Decoction Combined with Recombinant Human Interferon α2b on MRI Imaging, Tumor Markers, and Immune Function in Patients with Renal Cell Carcinoma" was published in 2021. Journal: Evid Based Complement Alternat Med.

After treatment, the complete ablation zone showed iso-high signal on T1WI in the treatment group. The signal intensity tended to be lower than before treatment, showing a high level of low-confounding signal. The T2WI fat suppression image showed low signal in the ablation zone. The residual cavity shadow left by the ablation antenna was a strip of high signal. After treatment, the ablation zone of the T2WI fat suppression image showed a mixed signal dominated by low signal, and the ablation zone gradually shrank. The signal had a tendency to increase unevenly, which was manifested as a mixed signal (Tables 2 and 3).

### 3.2. Observation of Recent Objective Curative Effect

The objective response rate (CR + PR) of the treatment group and the control group was 23.53% and 14.71%%, respectively. The disease control rate (CR + PR + SD) was 55.88% and 41.18%, respectively. There was no statistically significant difference in the objective efficacy between the treatment group and the control group (*P* > 0.05, Table 4).

### 3.3. Improvement of Common Clinical Symptoms

As shown in Table 5, the symptoms of loose stools were significantly worsened after treatment in the control group (*P* < 0.01). The symptoms of dry mouth and throat improved after treatment in the control group (*P* < 0.05, Table 5). The symptoms of hematuria, fatigue, dry mouth and throat, and five upset fever in the treatment group were significantly improved after treatment (*P* < 0.05, Table 5). After treatment, the soft symptoms of lumbar creatine were significantly improved in the treatment group (*P* < 0.05, Table 5). Comparing the two groups after treatment, the symptoms of poor appetite and obesity in the treatment group were significantly lighter than those in the control group (*P* < 0.05, Table 5). Compared with the two groups after treatment, the fatigue symptoms of the treatment group were lighter than those of the control group (*P* < 0.05, Table 5).

### 3.4. Karnofsky Score

The Karnofsky score in the treatment group was significantly higher after treatment than before treatment (*P* < 0.05, Figure 1), indicating that Chinese herbal decoction combined with recombinant human interferon *α*2b can significantly improve the life quality of patients. The Karnofsky score in the control group was higher than that before the treatment (*P* < 0.05, Figure 1), indicating that recombinant human interferon *α*2b also can improve the life quality of patients. Compared with the two groups after treatment, the treatment group was better than the control group in the improvement of Karnofsky score (*P* < 0.05, Figure 1). These results show that the combination of Chinese medicine decoction combined with recombinant human interferon *α*2b can increase the Karnofsky score and improve the physical status of patients compared with the use of recombinant human interferon *α*2b alone.

The article "The Effects of Chinese Herbal Decoction Combined with Recombinant Human Interferon α2b on MRI Imaging, Tumor Markers, and Immune Function in Patients with Renal Cell Carcinoma" was published in 2021. Journal: Evid Based Complement Alternat Med.

### 3.5. Comparison of White Blood Cell and Neutrophil Test Results between the Two Groups of Patients before and after Treatment

Recombinant human interferon *α*2b is a first-line immune drug for the treatment of RCC. However, patients will suffer varying degrees of blood cell reduction as well as clinical manifestations [21]. These adverse symptoms will lead to the reduction of interferon dosage or even the discontinuation of the drug, which will have a certain impact on the standard treatment of RCC patients. Therefore, the changes in the levels of white blood cells and neutrophils between the treatment group and the control group were detected (Figures 2 and 3).

As shown in Figures 2 and 3, the recovery rate of white blood cells and neutrophils in the treatment group was significantly higher than that in the control group (*P* < 0.05). The results indicate that the number of white blood cells can increase after giving patients oral Chinese medicine decoction. The possible reason is that the drug can enhance bone marrow hematopoietic function after being absorbed by the intestine. By monitoring the number of white blood cells in patients, it is found that the drug can indeed increase the number of white blood cells in patients, but the increase in some patients is not obvious.

### 3.6. The Changes of Tumor Marker Levels in Patients before and after Treatment

Before treatment, there was no significant difference in the levels of tumor markers between the two groups (*P* > 0.05, Table 6). After treatment, the levels of NSE and *β*2-MG in the two groups were significantly reduced. The NSE values in the treatment group and the control group were significantly reduced after treatment (*P* < 0.05, Table 6). Compared with the two groups after treatment, the treatment group was better than the control group in reducing NSE levels (*P* < 0.05, Table 6). The *β*2-MG values in the treatment group and the control group were decreased after treatment (*P* < 0.05, Table 6). But after treatment, there was no significant difference in the reduction of *β*2-MG levels between the treatment group and the control group (*P* > 0.05, Table 6).

The article "The Effects of Chinese Herbal Decoction Combined with Recombinant Human Interferon α2b on MRI Imaging, Tumor Markers, and Immune Function in Patients with Renal Cell Carcinoma" was published in 2021. Journal: Evid Based Complement Alternat Med.

### 3.7. Changes in the Proportion of T-Lymphocyte Factor Subgroups of Patients before and after Treatment

The CD4+/CD8+ ratio after treatment in the control group was significantly higher than before treatment (*P* < 0.01, Figure 4). The CD3+ and CD4+ values were higher than before treatment (*P* < 0.05, Figure 4). The CD8+ value was lower than before treatment (*P* < 0.05, Figure 4). After treatment, the CD3+, CD4+, and CD4+/CD8+ ratios in the treatment group were significantly increased (*P* < 0.05, Figure 4), and the CD8+ value was significantly decreased (*P* < 0.05, Figure 4). After treatment, the increase in the ratio of CD4+/CD8+ in the treatment group was significantly better than that in the control group (*P* < 0.05, Figure 4). After treatment, the treatment group was better than the control group in increasing CD3+ and CD4+ values and decreasing CD8+ value (*P* < 0.05, Figure 4). These results indicate that Chinese herbal decoction can improve the immune function of patients.

### 3.8. Quality of Life Score

The scores of nauseas and vomiting, loss of appetite, and diarrhea in the control group were significantly higher than those before treatment (*P* < 0.05, Table 7), indicating that these 4 items all deteriorated significantly after treatment. The scores of physical functions, role function, and social function were all higher than those before treatment (*P* < 0.05, Table 7), indicating that all 3 items were improved after treatment. The score of dyspnea was higher than that before treatment (*P* < 0.05, Table 7), indicating that this item aggravated after treatment. The role function and emotional function of the treatment group were significantly higher than before treatment (*P* < 0.05, Table 7), indicating that these two items were significantly improved after treatment. Both physical function and social function were improved compared with before treatment (*P* < 0.05, Table 7). The scores of fatigue and insomnia were lower than before treatment (*P* < 0.05, Table 7). It shows that all 4 items are improved after treatment. Nausea, vomiting, and diarrhea were all higher than before treatment (*P* < 0.05, Table 7), indicating that these two items aggravated after treatment.

After treatment, symptoms such as fatigue and nausea and vomiting in the treatment group were significantly lighter than those in the control group (*P* < 0.05, Table 7). After treatment, the treatment group was better than the control group in improving the patient's role function (*P* < 0.05, Table 7). The symptoms of insomnia and appetite loss in the treatment group were lighter than those in the control group (*P* < 0.05, Table 7). The emotional function and overall health of patients in the treatment group were better than those in the control group (*P* < 0.05, Table 7).

The article "The Effects of Chinese Herbal Decoction Combined with Recombinant Human Interferon α2b on MRI Imaging, Tumor Markers, and Immune Function in Patients with Renal Cell Carcinoma" was published in 2021. Journal: Evid Based Complement Alternat Med.

## 4. Discussion

At present, the toxic and side effects of RCC biological treatment are relatively large. The use of traditional Chinese medicine has a certain effect on reducing its toxic and side effects [22]. Interferon *α*2b has obvious effects of antitumor, which can inhibit cell proliferation and improve the body's immune function. After interferon *α*2b binds to the cell surface receptors, it can significantly improve the immune function of the patient's body, enhance the phagocytosis of macrophages, and accelerate cell apoptosis [23, 24]. However, after the application of interferon, patients often have symptoms such as fever, chills, body aches, cytopenias, nausea, and indigestion in varying degrees, leading to a reduction in interferon dose or even withdrawal. Therefore, this study explored the efficacy of Lishen Huazhuo Decoction combined with biological therapy in the treatment of RCC patients.

In recent years, due to the strengthening of people's awareness of physical examination and the improvement of inspection equipment, the detection rate of RCC has increased year by year. Percutaneous thermal ablation guided by image (ultrasound, CT, MR) is affected by factors, such as the operator's technical level, the limitations of imaging technology, the size, shape, location, and adjacent relationship of the tumor in the actual operation. This may lead to incomplete ablation and recurrence, and the ablation effect directly affects the patient's prognosis and quality of life. Among them, MRI has high soft tissue resolution and can be used for multisequence, multiparameter, and multidirectional imaging. MRI also has a variety of functional imaging methods, such as perfusion weighted imaging (PWI), diffusion weighted imaging (DWI), and magnetic resonance spectroscopy (MRS). Therefore, MRI is widely used in the treatment of RCC.

The results of this study show that the treatment group has a significant effect compared with the control group (Figure 5). After treatment, the clarity of lesion boundaries and MRI T1WI tumor marker levels in the treatment group were significantly lower than those in the control group. The objective remission rate, improvement of common symptoms, Karnofsky score, quality of life score, white blood cell and neutrophil count, and T lymphocyte factor subgroup ratio were significantly higher than those of the control group.

## 5. Conclusion

In summary, the treatment of RCC patients with recombinant human interferon *α*2b plus Chinese medicine decoction has obvious antitumor effect. Its components can also enhance the body's immunity and hematopoietic function and can greatly reduce the adverse reactions caused by hormone therapy. Chinese medicine decoction improves the patient's immunity and enhances the immunosuppressive effect of interferon *α*2b. At the same time, Chinese medicine decoction reduces the toxic and side effects caused by the application of immunosuppressive agents, improves the patient's life quality, and reduces the incidence of related adverse reactions. Therefore, recombinant human interferon *α*2b plus Chinese medicine decoction has obvious clinical therapeutic effects and is worthy of application in clinical work. However, the regulatory mechanism of recombinant human interferon *α*2b plus Chinese medicine decoction still needs to be further explored.

The article "The Effects of Chinese Herbal Decoction Combined with Recombinant Human Interferon α2b on MRI Imaging, Tumor Markers, and Immune Function in Patients with Renal Cell Carcinoma" was published in 2021. Journal: Evid Based Complement Alternat Med.

## Figures and Tables

**Figure 1:** Comparison of Karnofsky scores between two groups of patients before and after treatment (*x* ± *s*). ^*∗*^*P* < 0.05 (compared with before treatment); ^#^*P* < 0.05 (compared with the control group).

**Figure 2:** Comparison of peripheral blood leukocytes and counts between the two groups. ^*∗*^*P* < 0.05 (compared with before treatment); ^#^*P* < 0.05 (compared with the control group).

**Figure 3:** Comparison of neutrophil counts in peripheral blood between the two groups. ^*∗*^*P* < 0.05 (compared with before treatment); ^#^*P* < 0.05 (compared with the control group).

**Figure 4:** The changes of patients' CD3+, CD4+, CD8+, and CD4+/CD8+ before and after treatment. ^*∗*^*P* < 0.05 (compared with before treatment); ^#^*P* < 0.05 (compared with the control group).

**Figure 5:** The graphical abstract.

**Table 1:** Comparison of general information between the control group and the treatment group (*n* = 34).

Features		Control group	Treatment group

Age		58.97 ± 12.33	60.23 ± 13.79
Male/female		19/15	20/14
Karnofsky score		75.37 ± 7.324	73.674 ± 3.086

Tumor location	Left	17	18
	Right	17	16

Robson tumor stage	I	11	11
	II	15	16
	III	8	7

Case classification	Clear cell carcinoma	17	16
	Granular cell carcinoma	10	10
	Papillary RCC	7	8

**Table 2:** MRI manifestations of patients in the control group (*n* = 34).

Tine	Enhanced scan		
	Strengthened		No reinforcement
	Ring reinforcement	Irregularities or enhancement of marginal nodules	

Before treatment	19	5	10
After treatment	14	3	17

**Table 3:** MRI manifestations of patients in the treatment group (*n* = 34).

Tine	Enhanced scan		
	Strengthened		No reinforcement
	Ring reinforcement	Irregularities or enhancement of marginal nodules	

Before treatment	20	5	9
After treatment	12	2	20

**Table 4:** Comparison of short-term objective curative effect between the two groups of patients (case (%)).

Group	CR	PR	SD	PD	CR + PR	CR + PR + SD

Treatment group	2 (5.88%)	6 (17.65%)	11 (32.35%)	15 (22.12%)	8 (23.53%)	19 (55.88%)
Control group	1 (2.94%)	4 (11.76%)	9 (26.47%)	20 (58.82%)	5 (14.71%)	14 (41.18%)

The article "The Effects of Chinese Herbal Decoction Combined with Recombinant Human Interferon α2b on MRI Imaging, Tumor Markers, and Immune Function in Patients with Renal Cell Carcinoma" was published in 2021. Journal: Evid Based Complement Alternat Med.

**Table 5:** Comparison of common symptoms' improvement between the two groups of patients after treatment.

Common symptoms	Control group		Treatment group	
	Before	After	Before	After

Hematuria	1.54 ± 0.87	1.06 ± 0.89	1.58 ± 0.91	0.66 ± 0.51^*∗*^
Languid	1.63 ± 0.75	1.45 ± 0.63	1.64 ± 0.69	0.89 ± 0.33^*∗*^
Dry mouth and throat	1.86 ± 1.02	0.86 ± 0.42^*∗*^	1.98 ± 0.99	0.73 ± 0.72^*∗*^
Lumbar muscle soreness	1.54 ± 1.04	1.38 ± 0.92	1.59 ± 1.17	0.88 ± 0.93^*∗*^
Five upset fever	1.27 ± 0.85	1.03 ± 0.74	1.31 ± 0.89	0.59 ± 0.74^*∗*^
Abnormal stool	1.08 ± 0.43	1.36 ± 0.64	0.98 ± 0.39	1.64 ± 0.77^*∗*^
Poor appetite	1.61 ± 0.65	1.35 ± 0.21	1.63 ± 0.48	0.97 ± 0.37^*∗*#^

^*∗*^ *P* < 0.05 compared with this group before treatment; ^#^*P* < 0.05 compared with the control group.

**Table 6:** Changes of NSE, FERR, *β*2-MG, and CER levels of patients before and after treatment.

Indicator	Control group		Treatment group	
	Before	After	Before	After

NSE	19.38 ± 2.77	14.68 ± 2.53^*∗*^	19.29 ± 3.01	10.55 ± 2.13^*∗*#^
FERR	331.97 ± 86.03	268.43 ± 75.96	329.62 ± 90.31	265.27 ± 77.83
*β*2-MG	2714.85 ± 501.33	2035.17 ± 478.88^*∗*^	2702.31 ± 498.35	2006.64 ± 485.41^*∗*^
CER	3.10 ± 1.57	2.93 ± 2.01	3.08 ± 1.73	2.82 ± 1.78

^*∗*^Compared with before treatment, *P* < 0.05; ^#^compared with the control group, *P* < 0.05.

**Table 7:** Comparison of EORTC QLQ-C30 quality of life scores before and after treatment between the two groups.

Item	Control group		Treatment group	
	Before	After	Before	After

Functional subscale				
Physical function	45.75 ± 16.38	55.69 ± 18.35^*∗*^	45.77 ± 17.93	60.34 ± 19.81^*∗*^
Role function	59.43 ± 18.23	72.36 ± 20.19^*∗*^	60.44 ± 20.37	82.68 ± 21.52^*∗*#^
Cognitive function	58.03 ± 18.95	62.37 ± 20.06	57.91 ± 16.99	63.71 ± 18.82
Emotional function	51.36 ± 14.38	60.34 ± 19.97	54.39 ± 16.37	71.38 ± 21.79^*∗*#^
Social function	52.67 ± 16.57	64.77 ± 16.38^*∗*^	51.97 ± 14.39	67.03 ± 16.29^*∗*^

Symptom subscale				
Weak	44.07 ± 23.65	41.97 ± 19.06	43.98 ± 22.44	31.43 ± 18.73^*∗*#^
Pain	25.34 ± 19.25	32.76 ± 25.34	25.57 ± 21.79	29.14 ± 20.33
Nausea and vomiting	15.69 ± 12.12	47.38 ± 16.42^*∗*^	17.03 ± 5.63	32.58 ± 13.46^*∗*^
Breathing difficulties	38.23 ± 19.37	55.83 ± 28.71^*∗*^	38.04 ± 18.23	45.57 ± 23.31
Agrypnia	42.76 ± 21.83	48.21 ± 19.34	42.42 ± 21.39	24.39 ± 14.23^#^
Appetite loss	27.86 ± 19.34	57.14 ± 34.25^*∗*^	28.67 ± 20.47	40.26 ± 24.37
Constipation	37.45 ± 18.67	38.14 ± 20.00	36.71 ± 19.73	42.39 ± 21.37^*∗*^
Diarrhea	34.43 ± 22.37	59.37 ± 21.23	35.58 ± 19.19	54.38 ± 23.33
General health	55.27 ± 16.67	56.89 ± 20.41	55.83 ± 19.27	68.79 ± 20.43^#^

^*∗*^ *P* < 0.05, compared with this group before treatment; ^#^*P* < 0.05, compared with the control group.

The article "The Effects of Chinese Herbal Decoction Combined with Recombinant Human Interferon α2b on MRI Imaging, Tumor Markers, and Immune Function in Patients with Renal Cell Carcinoma" was published in 2021. Journal: Evid Based Complement Alternat Med.

## Data Availability

The datasets used during the present study are available from the corresponding author upon reasonable request.
